The article "Pars Plana Vitrectomy for a Sub-Internal Limiting Membrane Hemorrhage and Vitreous Hemorrhage Secondary to Dengue Fever: A Case Report" was published in 2022. Journal: Cureus.

# Pars Plana Vitrectomy for a Sub-Internal Limiting Membrane Hemorrhage and Vitreous Hemorrhage Secondary to Dengue Fever: A Case Report

**DOI:** 10.7759/cureus.25916

**Published:** 2022-06-13

**Authors:** Mohammad Ibn Abdul Malek, Jean Claude Niyonzima, Md. Arif Hayat Khan Pathan, Md. Mostafizur Rahman

**Affiliations:** 1 Vitreo-Retina and Uvea, Ispahani Islamia Eye Institute and Hospital, Dhaka, BGD

**Keywords:** ilm peeling, vitreous haemorrhage, pars plana vitrectomy, sub-internal limiting membrane haemorrhage, dengue fever

## Abstract

Although rare, dengue fever-associated ocular manifestations are a valid cause of visual impairment. Clinicians usually have a dilemma between vitrectomy and medical management if there is an associated vitreous hemorrhage. Vitrectomy has been rarely reported previously in the management of vitreous hemorrhage secondary to dengue fever.

We report a case of a young adult who presented with bilateral vitreous hemorrhages. The diagnosis of dengue was confirmed by serology and a typical epidemiological context. The patient presented already having undergone yttrium aluminum garnet (YAG) laser hyaloidotomy for preretinal hemorrhage in the other eye, with a subsequent vitreous spread of the hemorrhage. Vitrectomy with internal limiting membrane (ILM) peeling was performed for the affected eye and the visual acuity was fully regained after a few weeks.

Dengue fever can present with dense or sub-ILM hemorrhages. In our case, the vision quickly recovered after vitrectomy and ILM peeling. We, therefore, recommend early vitrectomy in cases with vitreous hemorrhage associated with sub-ILM involvement so as not to delay visual recovery.

## Introduction

Dengue fever is of public health concern worldwide [1]. According to WHO, tropical regions of Africa, South-east Asia, and South America are at increased risk with an estimated 50-100 millions of cases [2]. In Bangladesh, the peak incidence of outbreaks is said to coincide with the monsoon rainfall [3]. Two serotypes DEN1 and DEN2 are mostly isolated although the other two are also known to be prevalent in neighboring countries [4]. Efforts to curb the rapid progression of the disease by using a vaccine are underway [5-6]. Ocular manifestations of dengue fever have been reported in various countries of the endemic regions; sub-conjunctival, vitreous, preretinal and retrobulbar hemorrhages, maculopathy, vascular occlusions, and uveitis have been reported as the main clinical features [7-12]. The pathophysiology of ocular disease is yet to be agreed on, although immune-mediated reaction for the uveitis pathway and thrombocytopenia for the bleeding pathway have been postulated [8]. Recently, a theory proposed an increased level of hyaluronan to be responsible for vascular leakage and stated hyaluronan was an independent predictor for dengue fever severity and could be used to decide which patient to admit [13]. The treatment for ocular manifestations of dengue fever remains controversial. Steroids have been used by many authorities although there is no evidence to support their effectiveness [7]. Whereas sub-hyaloid and vitreous hemorrhage cases have been reported, little is known about vitrectomy in dengue fever associated vitreous hemorrhage. Two cases of pars plana vitrectomy were previously reported and none of them had sub-ILM hemorrhage as an indication but dense vitreous hemorrhage was the cited reason for vitrectomy [14-15]. In this case report, we share the complex diagnosis and management of the sub-ILM hemorrhage secondary to dengue fever.

The article "Pars Plana Vitrectomy for a Sub-Internal Limiting Membrane Hemorrhage and Vitreous Hemorrhage Secondary to Dengue Fever: A Case Report" was published in 2022. Journal: Cureus.

## Case presentation

A 34-year-old male patient presented on 2nd October 2019 to a vitreo-retina and uveitis specialist in Dhaka with complaints of blurring of vision in the recent days that seemed not to clear spontaneously. The patient denied having diabetes or hypertension. He also reported having a course of fever and headache that led to a serologic diagnosis of dengue fever. Besides the serologic diagnosis, the full blood count showed thrombocytopenia that persisted for a while (Table 1). Another systemic workup was unremarkable.

**Table 1:** Serological investigations. ALT, alanine transaminase

		Serological investigation			
Date	19/09/2019	21/09/2019	22/09/2019	25/09/2019	28/09/2019
Platelet count/cubic mm	140000	130000		45000	160000
ALT			196 U/L		41 U/L
Dengue NS1	Positive				

The presenting visual acuity was 1/60 in both eyes, the intraocular pressure was 15 mmHg in both eyes; on slit-lamp examination, there were no anterior segment abnormalities and the vitreous hemorrhage was noted in both eyes which was very mild in the right eye in association with a preretinal component involving the macula, while the dense vitreous hemorrhage made it impossible to examine the fundus in the left eye (Figure 1).

**Figure 1:** Color fundus photo at presentation. The figure shows right preretinal hemorrhage involving the macula and left eye vitreous hemorrhage.

The ultrasound exam of the left eye noted vitreous hemorrhage and queried a retinal detachment with regard to the 100% reflectivity spike on A-scan display (Figure 2).

**Figure 2:** Left eye B-scan ultrasound image. Note the hyperechogenic opacity in the posterior pole corresponding with the 100% reflectivity spike on A-scan.

Posterior yttrium aluminum garnet (YAG) laser hyaloidotomy was performed to free the macula in the right eye and nonsteroidal anti-inflammatory eye drops were instituted. The patient was reviewed on the 14th October. The exam noted persisting preretinal hemorrhage in the right eye despite the hyaloidotomy (Figure 3) whereas the vitreous hemorrhage was persistent in the left eye. The vision had improved to 6/18 in the right eye and remained 1/60 in the left eye. In view of the persisting vitreous hemorrhage, the patient was advised for pars plana vitrectomy and exploration.

The article "Pars Plana Vitrectomy for a Sub-Internal Limiting Membrane Hemorrhage and Vitreous Hemorrhage Secondary to Dengue Fever: A Case Report" was published in 2022. Journal: Cureus.

**Figure 3:** Right eye preretinal hemorrhage after posterior YAG laser capsulotomy. Note flesh blood migrating into the vitreous (arrow). YAG, yttrium aluminum garnet

Differential diagnosis

The diagnosis of vitreous hemorrhage as an ocular manifestation of dengue fever was rather straightforward in this patient particularly because he presented immediately after a course of fever and positive serology for dengue. However, in patients with dengue fever, vitreous hemorrhage can result from vascular occlusion or spontaneous bleeding. Moreover, the hemorrhage location can be intra-gel, sub-hyaloid, or sub-ILM each of them dictating a specific management plan. Intragel hemorrhages can be observed pending full resolution, with vitrectomy in persistent cases. Subhyaloid and sub-ILM hemorrhages are damaging due to the close proximity to the macula, and early vitrectomy is advocated [14]. Sub-ILM hemorrhages additionally require an ILM peel, as was needed in our case. In our patient, although the B-Scan suggested a retinal detachment, the intra-operative assessment concluded to a sub-ILM hemorrhage.

Management

Since the intra-gel vitreous hemorrhage in the left eye was dense to occlude the retinal assessment and did not improve over almost a month, a decision for pars plana vitrectomy for clearing the hemorrhage and retinal exploration was a logical next course of action. Intra-operatively, after a core vitrectomy and successful posterior vitreous detachment induction, it appeared there was a sub-ILM hemorrhage adjacent to the superior arcade. Staining with brilliant blue allowed the surgeon to peel the ILM and evacuate the hemorrhage. Two weeks postoperatively, the exam showed mild residual hemorrhage in the right eye and a clear vitreous cavity in the vitrectomized left eye (Figure 4).

**Figure 4:** Right eye shows cleared preretinal hemorrhage now located in the inferior quadrant vitreous (arrow). Left eye seen postoperatively.

Most importantly, the visual acuity had improved to 6/18. The vision continued to improve and was 6/6 as of the six-month follow-up.

## Discussion

Dengue fever related ocular manifestations have been reported especially in India and Brazil [6, 10]. The ocular findings are diversified but mainly hemorrhages, maculopathy, and uveitis are commonly discussed [8-10]. The diagnosis can be a challenge, especially in patients with systemic diseases like diabetes, hypertension, coagulation disorders, auto-immune diseases, and infections responsible for vasculitis retinae and secondary hemorrhage. Our patient was able to report promptly with all the medical records of his recent illness, rendering a more straightforward diagnosis. A good clinical history taking with specific questions or the knowledge of dengue fever in the region may be of utmost importance to link the current ocular conditions to dengue fever.

The article "Pars Plana Vitrectomy for a Sub-Internal Limiting Membrane Hemorrhage and Vitreous Hemorrhage Secondary to Dengue Fever: A Case Report" was published in 2022. Journal: Cureus.

Even with a good diagnosis, management challenges persist. In the literature, conservative measures and vitrectomy were used to manage the vitreous hemorrhage. Kumar and Ambiya performed a pneumatic sub-ILM hemorrhage displacement successfully [16]; their patient had a lighter vitreous hemorrhage that allowed them to visualize the macula unlike in our patient. Corticosteroids have been used in some cases in light of the immune-mediated disease pathway [17]. We presented a case of dense vitreous and sub-ILM hemorrhage that was managed surgically. This treatment option was motivated by the ultrasound image on one hand and the persistence of the hemorrhage over one month affecting the visual acuity. The literature is quiet to date on what are the indications for vitrectomy in dengue fever cases and the ophthalmologists have been left to judge on a case-by-case basis. A group of vitro-retinal (VR) ophthalmologists in the United Kingdom suggested early vitrectomy should be performed in fundus obscuring hemorrhages [15]. In our case, vitrectomy was very important to remove the sub-ILM hemorrhage that would have been very unlikely to clear spontaneously. The referral system and availability of surgical retina set-ups should be always taken into consideration when deciding to perform vitrectomy. With new vitrectomy equipment, we believe vitreous hemorrhage that affects seriously the vision could be treated surgically more often and timely than previously recommended. Our success story shows an impressive vision regained just two weeks after the surgery and the patient was happy to resume his duties without any delay.

## Conclusions

Although dengue fever ocular manifestations are rare, ophthalmologists seeing patients from outbreak regions or patients who recently visited such areas should have a high index of suspicion if they present with a recent history of fever and vitreous hemorrhage. If the vitreous hemorrhage is dense enough to affect the patient’s vision and daily activities or is located in the sub-ILM space, vitrectomy should be considered without delay.
